# Post Caesarean Section Deep Pelvic Abscess: CT Guided Transgluteal Drainage

**DOI:** 10.7759/cureus.21156

**Published:** 2022-01-12

**Authors:** Bharti Joshi, Maninder K Ghotra, Ujjwal Gorsi, Subhas Chandra Saha, Pooja Sikka

**Affiliations:** 1 Obstetrics and Gynaecology, Postgraduate Institute of Medical Education and Research, Chandigarh, IND; 2 Radiology, Postgraduate Institute of Medical Education and Research, Chandigarh, IND

**Keywords:** trans gluteal approach, percutaneous drainage, organ space surgical site infection, deep pelvic abscess, ct guided

## Abstract

Organ space surgical site infection (SSI), in itself, is a problematic condition for the surgeon and also adds pain and misery to the patient. If it happens along with deep pelvic collection, it further increases the risk of sepsis to the patient. Untreated abdominal or pelvic abscesses are associated with high mortality. This outcome is improved due to advances in image-guided percutaneous interventional techniques. The aim is to drain the collection with minimal morbidity to the patient. We report a case of deep surgical site infection following caesarean section in a COVID-19 positive patient managed with minimal intervention.

## Introduction

The pelvis is a frequent site of abscess formation, particularly in postoperative patients because it is the most dependent portion of the abdominal cavity. The infected fluid can easily collect there and become walled off. The deep pelvic collection is a part of the spectrum of organ space surgical site infection (SSI), which needs to be drained to prevent sepsis-related morbidity and mortality to the patient. Drainage of abdominal and pelvic abscesses via percutaneous route can be considered as an alternative to surgery and also provide time before surgery [1-3]. Percutaneous drainage of deep pelvic abscesses presents a unique challenge due to many anatomical obstacles which are at risk for injury during drainage. These include pelvic bones, iliac vessels, nerves, bowel, and urogenital organs. Thus, the imaging-guided approach is considered safe, which includes computed tomography (CT) guided or ultrasound-guided endocavitary drainage. A CT-guided transgluteal approach is a useful option when anterior or lateral approaches are not feasible. We hereby describe a postoperative case of caesarean section with deep pelvic abscess with wound SSI. The pelvic abscess was not drainable via vaginal approach due to the high-up location in the pelvis. Regarding the anterior approach, it was also not feasible as the uterus was stuck densely to the anterior abdominal wall with intervening bowel and urinary bladder. Thus, we approached the drainage of this patient via a CT-guided transgluteal method of pigtail placement. The patient responded well and was discharged on the fifth day.

## Case presentation

A 37-year-old antenatal gravida 4 para 2 with one living issue was admitted at 37 weeks of gestation with labor pains. She tested positive for COVID-19 on RT-PCR during routine testing, although there were no symptoms. Emergency caesarean section was done as she was not willing for the trial of labor after the previous caesarean section. A midline vertical incision was given; intraoperatively, she had dense adhesions. She received prophylactic antibiotics for three days and was discharged on the fourth day under stable conditions the with advice of home isolation. She had some discharge from the stitch line on the eighth day, for which she consulted at another centre of convenience, where the dressing was changed, and antibiotics were given. On day 12, she got her sutures removed and was diagnosed to have a deep surgical site infection, and was referred back to our institute. On examination, purulent discharge was coming through the wound. The sheath had given away, and the uterus was stuck at the incision site on the lower part; the sheath on the upper part of the incision site was intact. On per speculum examination, the vagina and cervix were healthy. Bi-manual examination revealed uterus was 14 weeks in size, non-tender, and bogginess was felt in the pouch of Douglas (POD). Ultrasonography of the whole abdomen showed an empty uterine cavity with 8 cm collection in POD, no free fluid in the abdominal cavity, and other organs were unremarkable. Wound debridement was done; the patient was started on intravenous antibiotics. The patient started to develop a high-grade fever. Contrast-enhanced CT abdomen showed around 8 cm collection in POD (Figure 1). Due to persistent fever, drainage was planned. Collection in POD should be amenable to be drained vaginally but was difficult as the collection was high up and anterior abdominal approach was not feasible because the uterus was stuck densely to the anterior abdominal wall, and there were intervening bowel loops in the urinary bladder. Therefore, transgluteal pigtail insertion was done under CT guidance. Under local anesthesia, the collection was approached through the left transgluteal approach with the patient in the prone position. Initial access was obtained using an 18 G Chiba needle through which 0.035-inch guidewire was passed into the pelvic collection using CT (Figure 1).

**Figure 1:** CT scan image shows initial needle placement in pelvic abscess via transgluteal approach.

After serial dilatation using fascial dilators, a 10 F pigtail catheter (Figure 2) was placed in the collection (Figure 3), and a drainage bag was attached. The wound manager was applied on the incision site. The patient became afebrile, and the pigtail was removed on the third day after radiological confirmation of no residual abscess, and the wound manager was removed on the fifth day. The daily dressing was continued, and the patient was discharged and followed up on an outpatient basis; later, resuturing was done. 

**Figure 2:** CT Scan image showing insertion of pigtail catheter after needle placement via transgluteal approach.

**Figure 3:** CT scan image showing track of pigtail catheter in sagittal section.

## Discussion

Percutaneous abscess drainage is the standard treatment in patients not requiring immediate surgery [4,5]. It can be done by different approaches like the anterior approach, which is considered the easiest one, but this approach may not be feasible in a few cases like our index patient. Therefore, other alternative roots like the vaginal approach through the posterior vaginal fornix, transgluteal approach, paracoccygeal-infragluteal approach for presacral abscesses, and transrectal approach used for perirectal abscess. The transgluteal approach, as used in our patient, is a safe and effective alternative to the anterior approach. To avoid complications and to plan safe access, the transgluteal approach requires precise anatomical knowledge of the pelvic region. Thus, to get a better spatial resolution for accurate localization of the collection and detection of adjacent neurovascular structures, it is usually performed under CT guidance [6]. Various landmarks are used on axial CT scans for transgluteal drainage. These include the sacrospinous ligament, piriformis muscle, sacral plexus, sciatic nerve, and gluteal vessels. In the transgluteal approach, the needle is directed caudal to the sacrospinous ligament, and it passes through the greater sciatic foramen, which involves the insertion of the catheter as close as possible to the sacrum to prevent injury to the rectum and at the level of the sacrospinous ligament. This infra-piriformis approach prevents transgression of the sciatic nerve, the sacral plexus, and the gluteal vessels. Another alternative to this infra-piriformis approach is the transpiriformis approach. For these approaches, the patient is placed in a ventral or lateral decubitus position. A review of the literature showed various case reports with successful drainage of transgluteal percutaneous drainage. This approach was first described in Butch et al.'s [7] report on 19 cases of pelvic abscess drainage. The largest evaluation of the transgluteal approach, including 154 cases of CT-guided transgluteal percutaneous drainage procedures in 140 patients, was reported recently by Harisinghani et al. [8], where complete resolution of abscesses was reported in 97.4%. This approach is associated with a significant drawback of patient discomfort [9]. Other rare complications associated with the transgluteal approach are pelvic haemorrhage, nerve injury, or the formation of large gluteal abscesses [10]. Thus, CT-guided transgluteal drainage of abdominal or pelvic abscesses provides a better alternative for those patients who cannot undergo immediate surgery. 

## Conclusions

In conclusion, the percutaneous CT-guided transgluteal approach is a simple, safe, well-tolerated, effective procedure for the treatment of deep pelvic abscesses that are inaccessible with an anterior approach. Infra-piriformis approaches are preferred to decrease the incidence of pain and neurovascular complications. Thus, transgluteal CT-guided drainage constitutes a useful alternative to endo cavitary drainage. This approach should be considered as the first-line intention for the treatment of deep pelvic abscesses.
